# Hyperglycemia Induces Toll-Like Receptor-2 and -4 Expression and Activity in Human Microvascular Retinal Endothelial Cells: Implications for Diabetic Retinopathy

**DOI:** 10.1155/2014/790902

**Published:** 2014-12-31

**Authors:** Uthra Rajamani, Ishwarlal Jialal

**Affiliations:** ^1^Laboratory for Atherosclerosis and Metabolic Research, Division of Endocrinology, Diabetes and Metabolism, Department of Pathology, University of California Davis Medical Center, Research Building 1, Room 3000, 4635 Second Avenue, Sacramento, CA 95817, USA; ^2^Veterans Affairs Medical Center, Mather, CA 95655, USA

## Abstract

Diabetic retinopathy (DR) causes visual impairment in working age adults and hyperglycemia-mediated inflammation is central in DR. Toll-like receptors (TLRs) play a key role in innate immune responses and inflammation. However, scanty data is available on their role in DR. Hence, in this study, we examined TLR2 and TLR4 mRNA and protein expression and activity in hyperglycemic human retinal endothelial cells (HMVRECs). HMVRECs were treated with hyperglycemia (HG) or euglycemia and mRNA and protein levels of TLR-2, TLR-4, MyD88, IRF3, and TRIF as well as NF-*κ*B p65 activation were measured. IL-8, IL-1*β*, TNF-*α* and MCP-1, ICAM-1, and VCAM-1 as well as monocyte adhesion to HMVRECs were also assayed. HG (25 mM) significantly induced TLR2 and TLR4 mRNA and protein in HMVRECs. It also increased both MyD88 and non-MyD88 pathways, nuclear factor-*κ*B (NF-*κ*B), biomediators, and monocyte adhesion. This inflammation was attenuated by TLR-4 or TLR-2 inhibition, and dual inhibition by a TLR inhibitory peptide as well as TLR2 and 4 siRNA. Additionally, antioxidant treatment reduced TLR-2 and TLR4 expression and downstream inflammatory markers. Collectively, our novel data suggest that hyperglycemia induces TLR-2 and TLR-4 activation and downstream signaling mediating increased inflammation possibly via reactive oxygen species (ROS) and could contribute to DR.

## 1. Introduction

Diabetes is a growing global epidemic affecting nearly 36 million people in USA alone and nearly 350 million worldwide. Diabetic retinopathy (DR) is the leading cause of vision impairment and blindness among working adults and afflicts around 30 percent of patients [1, 2]. Diabetes is a proinflammatory state characterized by elevated levels of C-reactive protein (CRP), inflammatory cytokines, chemokines, adhesion molecules, monocyte activity, and adipose tissue dysregulation [3–6]. Hyperglycemia in diabetes contributes to microvascular complications and reduction of glycemia reduces progression of microvascular disease such as retinopathy [1, 2]. Mechanisms that have been advanced to explain how hyperglycemia can induce DR include the polyol pathway, activation of protein kinase-C (PKC), increased oxidative stress, advanced glycation end product (AGE) formation, and increased inflammation [2, 7–9]. Also both increased oxidative stress and AGE receptor engagement can result in increased inflammation. Several studies have reported a role for inflammation in the development of DR [2, 7–10]. Inflammation results in an increase in NF-*κ*B activity, cytokines, chemokines, adhesion molecules, leukocyte adhesion, and leukostasis [2, 9, 10]. However the exact mechanism behind hyperglycemia-mediated inflammation leading to microvascular complications is unclear.

Toll-like receptors (TLRs) are pathogen-associated molecular pattern receptors and play a role in innate immune response [11, 12]. Their activation triggers a signaling cascade which results in the production of cytokines/chemokines, and so forth, thereby initiating an inflammatory response [11, 12]. Among the various TLRs, our group has shown increased TLR-2 and TLR-4 in type 1 and type 2 diabetes [13, 14]. Several other groups have also reported increased TLR expression and/or activity in muscle, B cells, and adipose tissue in diabetic patients [15, 16]. TLR-2 and TLR-4 have been shown to play an important role in atherosclerosis [16–18] and to be upregulated in patients with diabetic microvascular disease [19]. Furthermore genetic deficiency of TLR-2 and TLR-4 has resulted in an amelioration of diabetic nephropathy [20, 21]. However the role of TLRs in the pathogenesis of DR has not been explored. To this end, we determined the effect of hyperglycemia on TLR-2 and TLR-4 activity and on leukocyte adhesion in human microvascular retinal endothelial cells (HMVRECs) to gain insights for a role of TLRs in DR.

## 2. Methods

### 2.1. Human Microvascular Retinal Endothelial Cell Culture

Human microvascular retinal endothelial cells (HMVREC) were obtained from Cell Systems (Kirkland, WA, USA). The cells were isolated by elutriation and their endothelial nature was confirmed by positive immunofluorescence with vWF, CD31, and Dil-Ac-LDL uptake. There was no evidence of Muller cell (absence of CRALBP), pericyte as determined by absence of staining for *α*-smooth muscle actin, and the absence of glial cell contamination was determined by CD68 staining. They were maintained in endotoxin-free endothelial microvascular growth medium (Lonza, Walkersville, MD) supplemented with FBS and other growth factors at 37°C with 5% CO_2_ in attachment factor treated culture vessels. The cells, when confluent, were subsequently treated with 5.5 mM, 15 mM, and 25 mM glucose for 24 hours. During the course of HG treatment, the cells were maintained in basal endothelial growth media to avoid activation of TLRs by serum and other supplements. 19.5 mM mannitol/5.5 mM glucose was employed as an osmotic control.

### 2.2. Treatment

We employed the specific TLR-4 inhibitor, TAK 242 (0.5 *μ*M and 1 *μ*M) (Calbiochem, MA, USA), TLR-2 neutralizing antibody (100 nM and 200 nM) (Abcam, MA, USA), and TLR-2 and TLR-4 inhibitory peptide (TIP) (25 *μ*M and 50 *μ*M) (Imgenex, CA, USA) to test the effect of TLR inhibition on HG-mediated effects. Additionally, siRNA for TLR-2 and TLR-4 were employed. Antioxidants apocynin (Sigma, MO, USA) and N-acetyl cysteine (NAC) (Sigma, MO, USA) were employed to study the role of oxidative stress in TLR activation.

Subsequently, the cell supernatants and cell lysates were collected for assays and western blots. Additionally, nuclear extracts were separately collected for NF-*κ*B p65 assay.

### 2.3. siRNA Transfection

Prevalidated TLR-2 and TLR-4 small interfering RNA (siRNA) were obtained from Santa Cruz Biotechnology (Dallas, TX). HMVRECs were treated with 0.75 *μ*g siRNA for 18–24 hours in transfection media. The cells were replaced in complete media and allowed to settle for 24 hours. Subsequently cells were serum starved for 2 hours and HG treatments given as explained above.

### 2.4. Western Blot

Cell lysates (50 *μ*g protein) were resolved, transferred, and probed with TLR-4, TLR-2, myeloid differentiation factor 88 (MyD88), TRIF, and IRF3 antibodies as described previously [22]. Stripped membranes were used for *β*-actin as a loading control. Representative blots from four different experiments were used for analysis and in figures a representative blot is shown.

### 2.5. PCR

RNA from treated HMVRECs was extracted using trizol (Invitrogen, Carlsbad, CA). RT-PCR was performed using primers specific for TLR-2 and TLR-4 (InvivoGen, San Diego, CA), with glyceraldehyde-3-phosphate dehydrogenase (GAPDH) as control (R&D Systems, Minneapolis, MN). Band intensities were determined using ImageJ. TLR-2 and TLR-4 mRNA was expressed as a ratio of GAPDH as described previously [13, 22].

### 2.6. ELISA

Interleukin- (IL-) 1*β*, IL-8, tumor necrosis factor- (TNF-) *α*, monocyte chemoattractant protein- (MCP-) 1, vascular cell adhesion molecule- (VCAM-) 1, and intracellular adhesion molecule- (ICAM-) 1 were measured in the supernatants of HMVRECs by ELISA (Life Technologies, Grand Island, NY), as reported previously [23] and NF-kB p65 was measured in nuclear extracts (Active Motif, Carlsbad, CA) [22].

### 2.7. Endothelial Cell Adhesion Assay

HMVREC monolayers were cultured and treated as above. THP-1 cells were loaded with fluorescent CFDA-SE (carboxyfluorescein diacetate-succinimidyl ester) dye as described previously [24] for 30 minutes at 37°C. The labeled THP-1 cells were added to confluent HMVREC cells and incubated for 90 min. Thereafter the cells were gently washed using endothelial growth media and the number of bound cells were assayed by fluorescence excitation (485 nm) and emission (535 nm). TNF-*α* (10 ng/mL) served as the positive control.

### 2.8. ROS Measurement

Fluorescence microscopy was used to measure cellular ROS levels. Briefly, HMVRECs in culture were washed with warm PBS and treated with 25 *μ*M H_2_DCF-DA dye for 45 minutes at 37°C. Subsequently the cells were washed with PBS twice and immediately viewed using a FITC green filter (Ex 485/Em 535). ROS production in the cells was quantified by measuring the mean fluorescence intensity of at least 10 cells per image.

### 2.9. Statistical Analysis

Results from the experimental studies were reported as mean ± SD. Differences were analyzed by ANOVA with Newman-Keuls post hoc analyses. A probability value of *P* < 0.05 was considered significant. All statistical analyses were performed using GraphPad Prism Software (San Diego, CA).

## 3. Results

### 3.1. High Glucose Increases TLR-4 and TLR-2 Expression

HMVRECs were exposed to 5.5 mM (normal glucose), 15 mM, and 25 mM (HG) for 24 hours and mRNA expression and protein levels of TLR-2 and TLR-4 were determined. We observed that both 15 mM and 25 mM glucose treatments significantly increased TLR-4 (Figure 1(a)) and TLR-2 (Figure 1(c)) mRNA expression compared to 5.5 mM glucose (*P* < 0.01, *n* = 5). We did not observe any mRNA changes in TLR-2 or TLR-4 expression with the osmotic control of 19.5 mM mannitol/5.5 mM glucose compared to 5.5 mM glucose, suggesting that this increase in TLR-2 and TLR-4 expression is not an osmotic effect.

TLR-2 and TLR-4 protein levels in the normal and HG experiments were quantitated by western blots. High glucose (15 mM and 25 mM) increased TLR-2 and TLR-4 protein levels significantly (*P* < 0.05, *n* = 5) compared to normal glucose and mannitol consistent with our mRNA data (Figures 1(b) and 1(d)). It was also noted that 25 mM glucose treatment resulted in a greater increase in expression and receptor protein abundance compared to 15 mM glucose.

### 3.2. TLR Downstream-Signaling via MyD88 and Non-MyD88 Pathways

TLR-4 is known to signal via both MyD88 and non-MyD88 pathways while TLR-2 signals through the MyD88 pathway only [11, 12, 16]. Hence we measured signaling mediators of both MyD88 and non-MyD88 pathways since we showed that high glucose upregulates both TLR-2 and TLR-4. HG significantly induced MyD88, TRIF, and IRF3 suggesting that both MyD88 dependent and independent pathways are activated (Figure 2). Furthermore, high glucose (15 mM and 25 mM) also increased NF-*κ*B activity as evident from an increase in nuclear p65 compared to the normoglycemic control (*P* < 0.001, *n* = 5). With increases in TLR-2 and TLR-4 protein and NF-*κ*B activity, we also quantitated secreted inflammatory biomediators.

### 3.3. High Glucose Increases Circulating Biomediators of Inflammation

Secreted inflammatory biomediators IL-1*β*, IL-8, TNF-*α*, and MCP-1 were also increased significantly in 15 mM and 25 mM treatment with 25 mM treatment showing significantly higher induction compared to 15 mM (Figure 3).

### 3.4. High Glucose Increases Monocyte Adhesion

HG treatment resulted in increased secretion of the cell adhesion molecules (CAMs), ICAM-1, and VCAM-1. Endothelial cell adhesion assay measuring monocyte adhesion to HMVRECs also showed that there was increased monocyte adhesion with high glucose (Figure 4).

### 3.5. TLR-4/2 Inhibition Attenuates High Glucose-Mediated Inflammation

Since we have shown an increase in both TLR-2 and TLR-4 with high glucose, we next tested the relative contributions of these receptors to the increased inflammation including monocyte adhesion. The high glucose mediated increase in inflammatory biomediators such as IL-8, TNF-*α*, and MCP-1 were significantly attenuated on treatment with TAK 242, a small molecule specific inhibitor of TLR-4 adaptor protein-protein interaction and signaling [25]. It binds to TLR-4's intracellular domain at the cysteine-474 [26]. We employed 0.5 *μ*M and 1.0 *μ*M for TLR-4 inhibition and both concentrations (0.5 *μ*M and 1.0 *μ*M) attenuated TLR-4 signaling with 1.0 *μ*M showing more potent attenuation compared to 0.5 *μ*M (Figure 5(a)). Similarly both concentrations of TAK 242 decreased high glucose-mediated increases NF-*κ*B p65 activity, ICAM-1, and VCAM-1 and monocyte adhesion to HMVRECs (Figure 5(b)).

We next employed TIRAP inhibitory peptide (TIP) which is a TIRAP (toll-interleukin 1 receptor (TIR) domain adaptor protein) decoy protein that blocks both TLR-2 and TLR-4 signaling by interfering with signaling complex assembly [27]. Similar to TAK 242 treatment, TIP also significantly inhibited high glucose induced biomediator secretion (IL-8, TNF-*α*, and MCP-1) with more inhibition seen with 50 *μ*M concentration (Figure 6(a)). Also TIP treatment decreased high glucose induced nuclear p65 activity, ICAM-1, and VCAM-1 and monocyte adhesion to HMVRECs (Figure 6(b)).

We also employed a TLR-2 neutralizing antibody to inhibit TLR-2 signaling since there is no available small molecular inhibitor. Compared to high glucose, the TLR-2 neutralizing antibody significantly attenuated biomediator secretion (IL-8, TNF-*α*, and MCP-1) compared to high glucose at both concentrations (100 nM and 200 nM) with more inhibition seen with 200 nM concentration (Figure 7(a)). Nuclear p65, ICAM-1, and VCAM-1 levels as well as monocyte adhesion were significantly decreased by TLR-2 neutralizing antibody compared to high glucose (Figures 7(a) and 7(b)). We also employed an irrelevant control antibody and observed that it did not result in any significant inhibition in any of the biomediators measured.

Small interfering RNA (siRNA) against TLR-2 and TLR-4 resulted in at least 50% knockdown of the respective receptors as determined by western blotting for receptor levels (data not shown). In agreement with the above data, siRNA for both TLR-2 and TLR-4 also showed decreases in NF-*κ*B p65 as well as in secreted inflammatory biomediators such as TNF-*α* and IL-8 (Figure 8). In addition, increased THP-1 adhesion due to HG was also significantly reduced by siRNA treatment which further confirms our previous inhibitor studies.

### 3.6. High Glucose Mediated ROS Activates TLR-2 and TLR-4

Previously it has been shown that ROS is important in the induction of TLRs in monocytes [22]. HG treatment showed significant increases (approximately 2.5fold) in ROS levels as shown by H_2_DCFDA staining while both apocynin and NAC significantly lowered ROS levels (Figure 9). These changes in ROS were paralleled by an increase in both TLR-2 and TLR-4 mRNA expression and protein levels that were reduced with the inhibitors (Figure 9). There was almost a 1.6-fold increase in TLR-4 protein levels and a 2-fold increase in TLR-2 protein levels which were reduced to near normal levels by the antioxidants apocynin and NAC. HG-mediated increases in NF-*κ*B p65 levels were also attenuated significantly by both antioxidants (Figure 9). However it was noted that both apocynin and NAC showed similar decreases in ROS levels indicating that HG induces superoxide predominantly and that the TLR-2 and TLR-4 related effects observed could be mainly due to superoxide.

## 4. Discussion

Diabetic retinopathy (DR) is a chronic low-grade inflammatory disease of the retinal microvasculature [28]. Chronic inflammatory features such as increased microvascular permeability, leukostasis [29, 30], cytokine, chemokine, adhesion molecule expression [31], and neovascularization [32] are seen in DR. Several studies have implicated increased inflammation in DR [9, 10, 33, 34].

The primary aim of the present study was to determine the role of the pathogen recognition receptors, toll-like receptors (TLRs) specifically TLR-2 and TLR-4 in DR by investigating TLR activity in a pivotal cell in the pathogenesis of DR, that is, retinal ECs [2, 9, 28]. In this study we observe that both TLR-2 and TLR-4 were significantly increased in HMVREC by HG compared to normoglycemia. This observation is in agreement with previous reports from our group and others demonstrating increased expression and activity of TLR-2 and TLR-4 in monocytes, muscle, and adipose tissue of diabetic patients as we reviewed previously [16]. However it is the first report on TLR demonstration on microvascular endothelium that is increased with hyperglycemia. TLR-2/4 mediated MyD88 pathway was upregulated as shown by increased MyD88 protein levels and nuclear p65. Additionally, TLR-4-mediated Non-MyD88 pathway was also activated as indicated by the increased protein levels of TRIF and IRF3. These findings are in line with previous studies implicating hyperglycemia in renal microvascular complications. Kaur et al. reported increased TLR-4 expression and activity under hyperglycemic in renal mesangial cells incriminating TLR-4 in contributing to diabetic nephropathy [35]. Lin et al. showed increased TLR-4 expression under hyperglycemic conditions in human proximal tubular epithelial cells pointing towards a role for TLR-4 in tubulointerstitial inflammation in diabetic nephropathy [21]. We now extend these findings to a crucial cell in DR, the HMVRECs by showing increased TLR2 and 4 activity and biomediator release.

In this study we also show high glucose-mediated increases in inflammatory cytokines/chemokines such as IL-8, IL-1*β*, MCP-1, and TNF-*α*. It seems plausible that TLR-4/2 promotes inflammation, abnormal endothelial cell function in the retina, and retinal endothelial cell damage in DR. Previous studies suggest that oxidative stress appears to mediate the upregulation of TLRs under hyperglycemic conditions [22, 36]. Dasu et al. demonstrated in human monocytes that high glucose activated TLR2 and TLR4 expression, induction of MyD88, and non-MyD88-mediated signaling and NF-*κ*B activity. This effect appeared to be mediated via PKC activation of NADPH oxidase [22]. Another group also showed that knockout of the P47phox subunit of NADPH oxidase prevented upregulation of both TLR2 and TLR4 in diet-induced obesity [36].

Kowluru and Abbas showed elevated superoxide levels in retina of diabetic rats as well as retinal cells incubated in HG [37]. They also showed that antioxidant defense is diminished in diabetic retinae [38, 39]. Also Safi et al. using identical HMVRECs showed that high glucose induced both increase in biomarkers of oxidative stress and apoptosis [40]. However Busik et al. showed that HG did not stimulate endogenous ROS in retinal endothelial cells [41]. Furthermore, Busik et al. attributed HG-mediated retinal endothelial injury to cytokines released by other cells such as Muller cells and not directly to HG. However we have confirmed in our culture of HMVRECs the absence of other cells types such as Muller cells, pericytes (*α*-smooth muscle actin), or microglia (CD68) using immunofluorescence staining (data not shown) and hence can attribute the effects observed in HMVRECs. In our report on HMVRECs we show that high glucose induces ROS and both TLR2 and TLR4. Furthermore antioxidants, apocynin, and NAC reduced both ROS and TLR2 and TLR4 with a reduction in downstream signaling.

We further probed effects of HG by measuring adhesion molecules alongside performing monocyte adhesion assay as a measure of leukostasis, another important feature of DR. Several previous studies incriminate CAMs and cell adhesion in DR. Miyamoto et al. convincingly showed a role for increased ICAM-1 in leukostasis within retinal vessels of STZ-induced diabetes by demonstrating that a monoclonal antibody to ICAM-1 decreases both retinal leukostasis and vascular leakage [42]. Joussen et al. [34] showed that diabetic mice deficient in ICAM-1 or its ligand, CD18, were afforded protection from early features of DR including leukostasis, pericyte loss, and increased permeability. Meleth et al. reported that diabetic patients exhibit elevated levels of serum inflammatory markers including adhesion molecules compared to nondiabetic controls. They showed increased levels of RANTES, MCP-1, ICAM-1, VCAM-1, and VEGF additionally reporting that the levels of these cytokines were directly proportional to the severity of retinopathy [33]. In the current study we report that, in HMVRECs, there is an increase in adhesion molecules such as ICAM-1 and VCAM-1 and increased monocyte adhesion under hyperglycemic conditions, which is in agreement with previously published literature providing further validation for the model studied in this report. In contrast to our findings Vagaja et al. [43] showed that in hyperglycemic mice the classic ligand for TLR4, lipopolysaccharide, significantly reduced leukostasis but exacerbated two key features of DR, namely, injury to the endothelial cells and thinning of the retina. It needs to be pointed out that the TLR4 pathway (TLR-4 protein and downstream signaling) was not explored in this study. Moreover LPS treatment was only for 24 hours explaining their paradoxical finding with respect to leukostasis, since study duration needs to be several months in order to appreciate the pathology of DR [34].

Interestingly, the use of TAK 242, a specific small molecule inhibitor to TLR4, significantly attenuated the abovementioned increases in biomediators. TAK-242 (resatorvid) is a specific inhibitor of TLR-4 signaling that inhibits the production of TLR-4-triggered inflammatory mediators by binding to the intracellular domain of TLR4 [25, 26]. This synthetic inhibitor blocks TLR-4's intracellular domain TIR (toll/IL-1 receptor) [25, 26]. It impairs TLR-4's ability to associate with adaptor molecules, namely, TIRAP (MyD88 pathway) and TRAM (TIR-domain-containing adapter-inducing interferon-*β*-related adaptor molecule) (non-MyD88 pathway), blocking subsequent signal transduction. In this study we report TAK-242-mediated attenuation of inflammatory biomediators such as IL-8, IL-1*β*, TNF-*α*, and MCP-1 and NF-*κ*B activity in HG treated HMVRECs. These results clearly demonstrate that with high glucose the increases in p65 NF-*κ*B and inflammatory biomediators could be the result, in part, of an increase in TLR-4 signaling. Several studies have suggested a role for TLR-4 in HG mediated increased inflammation. Devaraj et al. showed in a STZ-diabetic TLR-4 knockout mouse model that there were reduced levels of MyD88, TRIF, and IRF3 and decreased NF-*κ*B activity compared to wild type diabetic mice [44]. Additionally they also showed reduced biomediator release (IL-1*β*, IL-6, IL-8, MCP-1, Interferon-*β*, and TNF-*α*) in diabetic TLR-4KO compared to diabetic wild type. Using a TLR-4 mutant mouse that impairs signal transduction, the investigators showed that TLR-4 signaling is involved in retinal damage and inflammation triggered by ischemic injury in a nondiabetic model [45]. Our data with TAK 242 further confirms the role of TLR-4 in inflammation and extends it to the diabetic retinal microcirculatory milieu.

Furthermore, TAK 242 treatment attenuates ICAM-1 and VCAM-1 levels in HG treated HMVRECs and shows a decrease in monocyte adhesion. Our findings in this study support previous reports that TLR-4 mediated ICAM-1 expression is attenuated with TLR-4 inhibition thus confirming TLR-4s' role in cell adhesion also in a retinal microvascular environment. Hence our study not only further strengthens the role of TLR-4 in HG mediated inflammation including leukocyte adhesion but also for the first time suggests a possible role in diabetic retinopathy.

We also employed a dual inhibitor, to both TLR-2 and TLR-4 to further elucidate the contributions of TLR-4 and TLR-2, using TIRAP inhibitory peptide (TIP), which is known to be an inhibitor of both TLR-2 and TLR-4 receptors. The TIRAP inhibitory peptide used in our study is a TR6 with a peptide sequence PGFLRDPWCKYQML. Couture et al. demonstrated that TIRAP inhibitory peptide TR6 significantly inhibits MyD88 recruitment in both TLR-2 and TLR-4 receptors. Additionally MyD88-independent pathway was also inhibited by TIP and the authors suggest that adaptor protein recruitment might occur sequentially at different cellular locations and controlled by TLR-4 trafficking [27]. The addition of TIP attenuated inflammatory cytokine secretion as measured by IL-8, TNF-*α*, and MCP-1 levels showed decreased NF-*κ*B p65 activation and decreased levels of ICAM-1 and VCAM-1 accompanied by decreased monocyte adhesion compared to HG treatment. Although TIP inhibits both TLR-2 and TLR-4, the level of attenuation of inflammatory cytokines or adhesion molecules was not significantly different from that of TAK 242. A possible explanation for this finding could be that although TLR-2 and TLR-4 expression is increased by high glucose, both inhibitors work by inhibiting the same downstream crucial signal transduction pathway, for example, NF-*κ*B. Tang et al. examined the role of deletion of MyD88 only from bone marrow derived cells on retinal pathology. They showed that MyD88 deletion in leukocytes inhibited diabetes-induced leukostasis, ICAM-1 expression, and retinal superoxide production. They also reported that deletion of TLR-2 and TLR-4 in leukocytes caused partial attenuation suggesting that both TLR2/4 and IL-1*β* signaling pathway play a role in diabetes-induced leukostasis and ICAM-1 expression and superoxide generation in retina [46]. Furthermore they showed that an agonist of TLR2 but not TLR4 induced both IL-8 and IL-6 in retina. Whilst they focused on the effect of leukocyte perturbations on retinal pathology their data support a role especially for TLR2 in DR.

TLR-2 inhibition using a TLR-2 neutralizing antibody once again attenuated inflammatory cytokine secretion as measured by IL-8, TNF-*α*, and MCP-1 levels, decreased nuclear p65, and decreased levels of ICAM-1 and VCAM-1 accompanied by decreased monocyte adhesion compared to HG treatment. TLR-2 has been implicated by some groups in diabetes-mediated microvascular complications. Devaraj et al. showed the involvement of TLR-2 in diabetic nephropathy. They utilized TLR-2 knockout animals and showed that absence of TLR-2 decreased proinflammatory state of diabetes alongside attenuation in inflammatory cytokines, albuminuria, podocyte effacement, and M1 macrophages in the kidney [20]. TLR2 signaling in intrinsic kidney cells has been shown to be required for the full development of inflammation, kidney damage, and fibrosis in diabetic nephropathy [47]. Collectively, these studies suggest a role for TLR-2 in HG mediated inflammation and support our current novel findings that TLR-2 inhibition attenuates inflammation and leukostasis in HMVRECs.

In an attempt to deduce the mechanism behind HG mediated activation of TLR-2 and TLR-4 in HMVRECs, we found that high glucose-mediated increase in ROS levels was associated with an increase in both TLR-2 and TLR-4 mRNA and protein expression as well as nuclear p65 activation. Several studies have shown the involvement of NADPH oxidase (Nox) in HG mediated ROS production in endothelial cells. Taye et al. showed increased expression of Nox subunits p47 (phox) and Nox 2 under high glucose in human umbilical artery endothelial cells [48]. The link between HG, Nox, and TLRs in monocytes was previously demonstrated by our group [22]. In the current study we show a link between HG and Nox using apocynin, an NADPH oxidase inhibitor, which attenuated ROS levels significantly proving that the ROS produced is by Nox predominantly. In addition, we make the novel finding in HMVRECs that apocynin treatment showed decreases in TLR-2 and TLR-4 mRNA and protein levels. We have previously shown in monocytes that HG mediated superoxide release is via PKC-*α* activation [22, 49]. Thallas-Bonke et al. showed in diabetic renal disease that PKC-*α* is a key mechanism for Nox activation [50]. Taken together these studies point towards Nox activation and subsequent superoxide in our setting being PKC-*α* mediated.

We also employed another antioxidant N-acetyl cysteine (NAC) which serves as a prodrug to L-cysteine that acts as a precursor for glutathione. NAC, similar to apocynin, decreased ROS levels as well as mRNA and protein levels of both TLR-2 and TLR-4. It was however noted that NAC treatment brought about a similar degree of change in TLR-2 and TLR-4 levels as apocynin. This goes on to further prove that, in our experimental setting, superoxide was the predominant ROS produced due to HG which activates TLR-2 and TLR-4 in the absence of TLR ligands such as bacterial endotoxins.

However we would also like to point out that although care was taken to avoid endotoxin contamination in the media the presence of small amounts of endotoxins in the cellular environment is possible given the fact that the cells were cultured in the presence of serum and other cellular supplements which could be sources of endotoxins. Also it needs to be pointed out that Morigi et al. have previously documented an increase in leukocyte adhesion and NF-kB activity with hyperglycemia in the absence of other agonists [51].

## 5. Conclusion

The current study sheds light on an area which has not been explored thus far, microvascular endothelial TLRs in DR. Our study clearly points towards a role for TLR-4- and TLR-2-induced inflammation in the genesis of DR. In addition to showing upregulation and increased activity of both TLR-2 and TLR-4 with HG, we also show using different inhibitors that we can attenuate the TLR-mediated increased inflammation. Additionally, we show that this TLR-2 and TLR-4 activation is ROS mediated, specifically Nox derived superoxide-mediated and that antioxidant treatment helped in abrogation of TLR activation. We make the novel observation that both TLR-2 and TLR-4 are induced by high glucose in microvascular retinal endothelial cells and could possibly contribute to DR by inducing increased inflammation. This report could prove an impetus for future studies testing the role of both TLR-4 and TLR-2* in vivo* in DR by using diabetic wild type and knockout mice or small molecule inhibitors.

## Figures and Tables

**Figure 1:** High glucose (HG) induces toll-like receptor-4 (TLR-4) and TLR-2: confluent HMVRECs were serum-starved for 2 hours and incubated for 24 hours with 5.5, 15, and 25 mM glucose or mannitol (M) 19.5 mM/5.5 mM glucose for 24 hours. Thereafter the cells were harvested for mRNA in trizol or protease inhibitor buffer for cell lysates. (a) High glucose induces TLR-4 mRNA expression in human microvascular endothelial cells (HMVRECs). Bar graphs representing hyperglycemia-induced TLR-4 mRNA expression normalized to GAPDH. ^*^ *P* < 0.001 versus control and ^†^ *P* < 0.01 versus 15 mM; (b) HG induces TLR-4 protein levels in HMVRECs. Bar graph representing TLR-4 protein levels normalized to *β*-actin. ^*^ *P* < 0.01 versus control, ^**^ *P* < 0.001 versus control, and ^†^ *P* < 0.001 versus 15 mM; (c) high glucose induces TLR-2 mRNA expression in HMVRECs. Bar graphs representing hyperglycemia-induced TLR-2 mRNA expression normalized to GAPDH. ^*^ *P* < 0.001 versus control and ^†^ *P* < 0.001 versus 15 mM; (d) HG induces TLR-2 protein levels in HMVRECs. Bar graph representing TLR-2 protein levels normalized to *β*-actin. ^*^ *P* < 0.05 versus control, ^**^ *P* < 0.01 versus control, and ^†^ *P* < 0.05 versus 15 mM.

**Figure 2:** High glucose induces both MyD88 and Non-MyD88 pathways: HMVRECs were incubated and treated with 5.5, 15, and 25 mM glucose and mannitol as described in Methods and legend of Figure 1 and protein lysates were harvested. (a) Western blots showing increased MyD88 protein levels normalized against *β*-actin. ^*^ *P* < 0.01 versus control and ^**^ *P* < 0.001 versus control. ^†^ *P* < 0.05 versus 15 mM, (b) increased nuclear p65 levels with HG treatment. ^*^ *P* < 0.001 versus control. ^†^ *P* < 0.05 versus 15 mM, (c) representative blots showing increased TRIF and IRF3 protein levels with HG. Blots are normalized against *β*-actin. TRIF: ^*^ *P* < 0.05 versus control; ^**^ *P* < 0.001 versus control; IRF3 ^*^ *P* < 0.01 versus control, ^**^ *P* < 0.001 versus control, and ^†^ *P* < 0.05 versus 15 mM.

**Figure 3:** High glucose induces increased inflammatory biomediator release: HMVRECs were incubated and treated with 5.5, 15, and 25 mM glucose and mannitol as described in Methods and legend of Figure 1. Thereafter cell supernatants were collected for ELISA. (a) IL-8, (b) IL-1*β*, (c) TNF-*α*, and (d) MCP-1 levels are increased under hyperglycemic conditions. ^*^ *P* < 0.001 versus controls and ^†^ *P* < 0.001 versus 15 mM.

**Figure 4:** High glucose induced cell adhesion: HMVRECs were incubated and treated with 5.5, 15, and 25 mM glucose and mannitol as described in Methods and legend of Figure 1. Thereafter cell supernatants were collected for ELISA. Adhesion assay is described in Methods section. (a) Increased ICAM-1 levels with HG. ^*^ *P* < 0.01 versus controls and ^**^ *P* < 0.001 versus controls, (b) increased sVCAM-1 levels with HG. ^*^ *P* < 0.001 versus controls; (c) cell adhesion assay showing increased cell adhesion with HG. ^*^ *P* < 0.001 versus control.

**Figure 5:** (a) TLR-4 inhibition by TAK 242 attenuates downstream inflammatory biomediators: HMVRECs were serum starved for 2 hours and treated with 0.5 and 1 *μ*M TAK-242 for 2 hours. Thereafter 5.5 and 25 mM glucose treatments were performed as described in Figure 3. (I) NF-*κ*B, (II) IL-8, (III) TNF-*α*, and (IV) MCP-1 levels are significantly decreased upon TLR-4 inhibition compared to HG treatment. ^#^ *P* < 0.001 versus control, ^*^ *P* < 0.001 versus 25 mM, and ^†^ *P* < 0.01 versus 0.5 *μ*M TAK242. (b) Cell adhesion molecules ICAM-1 and VCAM-1 attenuation upon TAK 242 treatment. HMVRECs were serum starved for 2 hours and treated with 0.5 and 1 *μ*M TAK-242 for 2 hours. Thereafter 5.5 and 25 mM glucose treatments were performed as described in Figure 4. Adhesion molecules (I) ICAM-1 and (II) VCAM-1 levels are significantly decreased upon TAK242 treatment. ^#^ *P* < 0.001 versus control and ^*^ *P* < 0.001 versus 25 mM. (III) Adhesion assay showing decreased cell adhesion with TLR-4 inhibition. ^#^ *P* < 0.001 versus control, ^*^ *P* < 0.01 versus 25 mM, and ^**^ *P* < 0.001 versus 25 mM.

**Figure 6:** (a) TLR-2/4 inhibition by TIP attenuates downstream inflammatory biomediators: HMVRECs were serum starved for 2 hours and treated with 25 and 50 *μ*M TIP for 2 hours. Thereafter 5.5 and 25 mM glucose treatments were performed as described in Figure 3. (I) NF-*κ*B, (II) TNF-*α*, (III) IL-8, and (IV) MCP-1 levels are significantly decreased upon TLR-2/4 inhibition compared to HG treatment. ^#^ *P* < 0.001 versus control, ^*^ *P* < 0.001 versus 25 mM, and ^†^ *P* < 0.01 versus 25 *μ*M TIP. (b) Cell adhesion molecules ICAM-1 and VCAM-1 attenuation upon TIP treatment. HMVRECs were serum starved for 2 hours and treated with 25 and 50 *μ*M TIP for 2 hours. Thereafter 5.5 and 25 mM glucose treatments were performed as described in Figure 4. Adhesion molecules (I) ICAM-1 and (II) VCAM-1 levels are significantly decreased upon TIP treatment. ^#^ *P* < 0.001 versus control and ^*^ *P* < 0.001 versus 25 mM. (III) Adhesion assay showing decreased cell adhesion with TLR-2/4 inhibition. ^#^ *P* < 0.001 versus control and ^*^ *P* < 0.01 versus 25 mM.

**Figure 7:** (a) TLR-2 inhibition by TLR-2 neutralizing antibody attenuates downstream inflammatory biomediators: HMVRECs were serum starved for 2 hours and treated with 100 and 200 nM TLR-2 neutralizing antibody for 2 hours. Thereafter 5.5 and 25 mM glucose treatments were performed as described in Figure 3. (I) NF-*κ*B, (II) TNF-*α*, (III) IL-8, and (IV) MCP-1 levels are significantly decreased upon TLR-2 inhibition compared to HG treatment. ^#^ *P* < 0.001 versus control, ^*^ *P* < 0.001 versus 25 mM, and ^†^ *P* < 0.01 versus 100 nM. (b) Cell adhesion molecules ICAM-1 and VCAM-1 attenuation upon TLR-2 neutralizing antibody treatment. HMVRECs were serum starved for 2 hours and treated with 100 and 200 nM TLR-2 neutralizing antibody for 2 hours. Thereafter 5.5 and 25 mM glucose treatments were performed as described in Figure 4. Adhesion molecules (I) ICAM-1 and (II) VCAM-1 levels are significantly decreased upon TLR-2 inhibition. ^#^ *P* < 0.001 versus control and ^*^ *P* < 0.001 versus 25 mM. (III) Adhesion assay showing decreased cell adhesion with TLR-2 inhibition. ^#^ *P* < 0.001 versus control and ^*^ *P* < 0.01 versus 25 mM.

**Figure 8:** siRNA for TLR-2 and TLR-4 attenuates downstream inflammatory biomediators: HMVRECs treated with 0.75 *μ*g siRNA for 18–24 hours in transfection media. The cells were replaced in complete media and allowed to settle for 24 hours. Subsequently cells were serum starved for 2 hours and HG treatments given as described in Figure 1. (a) NF-*κ*B, (b) TNF-*α*, and (c) IL-8. ^#^ *P* < 0.001 versus control and ^*^ *P* < 0.001 versus 25 mM; Sc: scrambled sense RNA.

**Figure 9:** Antioxidant treatment attenuates HG-mediated ROS and TLR-2 and TLR-4 activation: HMVRECs treated with apocynin (60 *μ*M) and N-acetyl cysteine (10 mM) and subsequently exposed to high glucose. (a) ROS measurement by H_2_DCFDA staining. ^#^ *P* < 0.001 versus control and ^*^ *P* < 0.001 versus 25 mM; (b) TLR-2 and TLR-4 protein levels measured using western blot. ^#^ *P* < 0.01 versus control and ^*^ *P* < 0.01 versus 25 mM; (c) TLR-2 and TLR-4 mRNA expression measured by PCR. ^#^ *P* < 0.01 versus control and ^#^ *P* < 0.05 versus 25 mM. (d) NF-*κ*B p65 measurement by ELISA, ^#^ *P* < 0.001 versus control and ^*^ *P* < 0.001 versus 25 mM.

## References

[1] Antonetti D. A., Barber A. J., Bronson S. K. (2006). Diabetic retinopathy: seeing beyond glucose-induced microvascular disease. *Diabetes*.

[2] Cheung N., Mitchell P., Wong T. Y. (2010). Diabetic retinopathy. *The Lancet*.

[3] Schram M. T., Chaturvedi N., Schalkwijk C. (2003). Vascular risk factors and markers of endothelial function as determinants of inflammatory markers in type 1 diabetes: the EURODIAB prospective complications study. *Diabetes Care*.

[4] Shanmugam N., Reddy M. A., Guha M., Natarajan R. (2003). High glucose-induced expression of proinflammatory cytokine and chemokine genes in monocytic cells. *Diabetes*.

[5] Devaraj S., Glaser N., Griffen S., Wang-Polagruto J., Miguelino E., Jialal I. (2006). Increased monocytic activity and biomarkers of inflammation in patients with type 1 diabetes. *Diabetes*.

[6] Devaraj S., Dasu M. R., Jialal I. (2010). Diabetes is a proinflammatory state: a translational perspective. *Expert Review of Endocrinology & Metabolism*.

[7] van Hecke M. V., Dekker J. M., Nijpels G. (2005). Inflammation and endothelial dysfunction are associated with retinopathy: the Hoorn Study. *Diabetologia*.

[8] Klein B. E. K., Knudtson M. D., Tsai M. Y., Klein R. (2009). The relation of markers of inflammation and endothelial dysfunction to the prevalence and progression of diabetic retinopathy: wisconsin epidemiologic study of diabetic retinopathy. *Archives of Ophthalmology*.

[9] Tang J., Kern T. S. (2011). Inflammation in diabetic retinopathy. *Progress in Retinal and Eye Research*.

[10] Tarr J. M., Kaul K., Chopra M., Kohner E. M., Chibber R. (2013). Pathophysiology of diabetic retinopathy. *ISRN Ophthalmology*.

[11] Akira S., Takeda K. (2004). Toll-like receptor signalling. *Nature Reviews Immunology*.

[12] Beutler B. (2004). Inferences, questions and possibilities in Toll-like receptor signalling. *Nature*.

[13] Devaraj S., Dasu M. R., Rockwood J., Winter W., Griffen S. C., Jialal I. (2008). Increased toll-like receptor (TLR) 2 and TLR4 expression in monocytes from patients with type 1 diabetes: further evidence of a proinflammatory state. *The Journal of Clinical Endocrinology & Metabolism*.

[14] Dasu M. R., Devaraj S., Park S., Jialal I. (2010). Increased Toll-Like Receptor (TLR) activation and TLR ligands in recently diagnosed type 2 diabetic subjects. *Diabetes Care*.

[15] Creely S. J., McTernan P. G., Kusminski C. M. (2007). Lipopolysaccharide activates an innate immune system response in human adipose tissue in obesity and type 2 diabetes. *American Journal of Physiology—Endocrinology and Metabolism*.

[16] Jialal I., Kaur H. (2012). The role of toll-like receptors in diabetes-induced inflammation: implications for vascular complications. *Current Diabetes Reports*.

[17] Michelsen K. S., Wong M. H., Shah P. K. (2004). Lack of toll-like receptor 4 or myeloid differentiation factor 88 reduces atherosclerosis and alters plaque phenotype in mice deficient in apolipoprotein E. *Proceedings of the National Academy of Sciences of the United States of America*.

[18] Mullick A. E., Tobias P. S., Curtiss L. K. (2005). Modulation of atherosclerosis in mice by Toll-like receptor 2. *The Journal of Clinical Investigation*.

[19] Devaraj S., Jialal I., Yun J.-M., Bremer A. (2011). Demonstration of increased toll-like receptor 2 and toll-like receptor 4 expression in monocytes of type 1 diabetes mellitus patients with microvascular complications. *Metabolism: Clinical and Experimental*.

[20] Devaraj S., Tobias P., Kasinath B. S., Ramsamooj R., Afify A., Jialal I. (2011). Knockout of toll-like receptor-2 attenuates both the proinflammatory state of diabetes and incipient diabetic nephropathy. *Arteriosclerosis, Thrombosis, and Vascular Biology*.

[21] Lin M., Yiu W. H., Wu H. J. (2012). Toll-like receptor 4 promotes tubular inflammation in diabetic nephropathy. *Journal of the American Society of Nephrology*.

[22] Dasu M. R., Devaraj S., Zhao L., Hwang D. H., Jialal I. (2008). High glucose induces toll-like receptor expression in human monocytes: mechanism of activation. *Diabetes*.

[23] Jialal I., Huet B. A., Kaur H., Chien A., Devaraj S. (2012). Increased toll-like receptor activity in patients with metabolic syndrome. *Diabetes Care*.

[24] Venugopal S. K., Devaraj S., Yuhanna I., Shaul P., Jialal I. (2002). Demonstration that C-reactive protein decreases eNOS expression and bioactivity in human aortic endothelial cells. *Circulation*.

[25] Matsunaga N., Tsuchimori N., Matsumoto T., Ii M. (2011). TAK-242 (resatorvid), a small-molecule inhibitor of Toll-like receptor (TLR) 4 signaling, binds selectively to TLR4 and interferes with interactions between TLR4 and its adaptor molecules. *Molecular Pharmacology*.

[26] Takashima K., Matsunaga N., Yoshimatsu M. (2009). Analysis of binding site for the novel small-molecule TLR4 signal transduction inhibitor TAK-242 and its therapeutic effect on mouse sepsis model. *British Journal of Pharmacology*.

[27] Couture L. A., Piao W., Ru L. W., Vogel S. N., Toshchakov V. Y. (2012). Targeting toll-like receptor (TLR) signaling by toll/interleukin-1 receptor (TIR) domain-containing adapter protein/MyD88 adapter-like (TIRAP/Mal)-derived decoy peptides. *Journal of Biological Chemistry*.

[28] Kern T. S. (2007). Contributions of inflammatory processes to the development of the early stages of diabetic retinopathy. *Experimental Diabetes Research*.

[29] Mathews M. K., Merges C., McLeod D. S., Lutty G. A. (1997). Vascular endothelial growth factor and vascular permeability changes in human diabetic retinopathy. *Investigative Ophthalmology and Visual Science*.

[30] Hikichi T., Fujio N., Akiba J., Azuma Y., Takahashi M., Yoshida A. (1997). Association between the short-term natural history of diabetic macular edema and the vitreomacular relationship in type II diabetes mellitus. *Ophthalmology*.

[31] Canataroglu H., Varinli I., Ozcan A. A., Canataroglu A., Doran F., Varinli S. (2005). Interleukin (IL)-6, interleukin (IL)-8 levels and cellular composition of the vitreous humor in proliferative diabetic retinopathy, proliferative vitreoretinopathy, and traumatic proliferative vitreoretinopathy. *Ocular Immunology and Inflammation*.

[32] Schroder S., Palinski W., Schmid-Schonbein G. W. (1991). Activated monocytes and granulocytes, capillary nonperfusion, and neovascularization in diabetic retinopathy. *American Journal of Pathology*.

[33] Meleth A. D., Agrón E., Chan C.-C. (2005). Serum inflammatory markers in diabetic retinopathy. *Investigative Ophthalmology and Visual Science*.

[34] Joussen A. M., Poulaki V., Le M. L. (2004). A central role for inflammation in the pathogenesis of diabetic retinopathy. *The FASEB Journal*.

[35] Kaur H., Chien A., Jialal I. (2012). Hyperglycemia induces toll like receptor 4 expression and activity in mouse mesangial cells: Relevance to diabetic nephropathy. *The American Journal of Physiology—Renal Physiology*.

[36] Chen J.-X., Stinnett A. (2008). Critical role of the NADPH oxidase subunit p47phox on vascular TLR expression and neointimal lesion formation in high-fat diet-induced obesity. *Laboratory Investigation*.

[37] Kowluru R. A., Abbas S. N. (2003). Diabetes-induced mitochondrial dysfunction in the retina. *Investigative Ophthalmology and Visual Science*.

[38] Kowluru R. A., Tang J., Kern T. S. (2001). Abnormalities of retinal metabolism in diabetes and experimental galactosemia. VII. Effect of long-term administration of antioxidants on the development of retinopathy. *Diabetes*.

[39] Kern T. S., Kowluru R. A., Engerman R. L. (1994). Abnormalities of retinal metabolism in diabetes or galactosemia: ATPases and glutathione. *Investigative Ophthalmology & Visual Science*.

[40] Safi S. Z., Qvist R., Yan G. O., Ismail I. S. (2014). Differential expression and role of hyperglycemia induced oxidative stress in epigenetic regulation of *β*1, *β*2 and *β*3-adrenergic receptors in retinal endothelial cells. *Acta Veterinaria Scandinavica*.

[41] Busik J. V., Mohr S., Grant M. B. (2008). Hyperglycemia-induced reactive oxygen species toxicity to endothelial cells is dependent on paracrine mediators. *Diabetes*.

[42] Miyamoto K., Khosrof S., Bursell S.-E. (1999). Prevention of leukostasis and vascular leakage in streptozotocin-induced diabetic retinopathy via intercellular adhesion molecule-1 inhibition. *Proceedings of the National Academy of Sciences of the United States of America*.

[43] Vagaja N. N., Binz N., McLenachan S., Rakoczy E. P., McMenamin P. G. (2013). Influence of endotoxin-mediated retinal inflammation on phenotype of diabetic retinopathy in Ins2Akita mice. *British Journal of Ophthalmology*.

[44] Devaraj S., Tobias P., Jialal I. (2011). Knockout of toll-like receptor-4 attenuates the pro-inflammatory state of diabetes. *Cytokine*.

[45] Dvoriantchikova G., Barakat D. J., Hernandez E., Shestopalov V. I., Ivanov D. (2010). Toll-like receptor 4 contributes to retinal ischemia/reperfusion injury. *Molecular Vision*.

[46] Tang J., Allen Lee C., Du Y. (2013). MyD88-dependent pathways in leukocytes affect the retina in diabetes. *PLoS ONE*.

[47] Ma J., Wu H., Zhao C. Y., Panchapakesan U., Pollock C., Chadban S. J. (2014). Requirement for TLR2 in the development of albuminuria, inflammation and fibrosis in experimental diabetic nephropathy. *International Journal of Clinical and Experimental Pathology*.

[48] Taye A., Saad A. H., Kumar A. H., Morawietz H. (2010). Effect of apocynin on NADPH oxidase-mediated oxidative stress-LOX-1-eNOS pathway in human endothelial cells exposed to high glucose. *European Journal of Pharmacology*.

[49] Dasu M. R., Devaraj S., Jialal I. (2007). High glucose induces IL-1*β* expression in human monocytes: mechanistic insights. *American Journal of Physiology—Endocrinology and Metabolism*.

[50] Thallas-Bonke V., Thorpe S. R., Coughlan M. T. (2008). Inhibition of NADPH oxidase prevents advanced glycation end product-mediated damage in diabetic nephropathy through a protein kinase C-*α*-dependent pathway. *Diabetes*.

[51] Morigi M., Angioletti S., Imberti B. (1998). Leukocyte-endothelial interaction is augmented by high glucose concentrations and hyperglycemia in a NF-kB-dependent fashion. *Journal of Clinical Investigation*.

